RETRACTED

# Construction of Community Life Service in the Sharing Economy Based on Deep Neural Network

**DOI:** 10.1155/2021/7703152

**Published:** 2021-09-11

**Authors:** Di Qu, Dianya Deng

**Affiliations:** South China University of Technology, Guangzhou 510640, Guangdong, China

## Abstract

Currently, the development of sharing economy and interconnection also has a profound impact on community life services. This study is based on the deep neural network theory, combined with the evolution mechanism of the commercial network of the community life service industry, link prediction theory, and the latest deep neural network algorithm, referring to the evolution model of merger and stripping, and the network structure is optimized on this basis. Through simulation experiments and result analysis, the model is used to deeply study the evolution trend and dynamics of the community life service business network from the perspective of quantitative analysis. Then the business network structure is optimized and development is promoted at the same time. At the same time, it can also upgrade those old scattered industries and provide theoretical and decision-making guidance for the future transformation and upgrading of the innovative community life service industry.

## 1. Introduction

In recent years, with the rapid development of sharing economy, bike sharing, online taxi booking, and other forms of new business have been also emerging. Platform enterprises effectively connect the supply and demand of the society, make idle resources have more effective use, and obtain rapid development with the outstanding advantages of price and service [1]. The development of sharing economy and interconnection also has a profound impact on community life services. The application system of community life service e-commerce and sharing economy has developed rapidly; “shared intelligent cabinet,” “vegetable through train,” and “community group buying” appear in the community business model [2]. The innovative community life service industry is gradually becoming the development trend of the future community life service industry through its advantages of innovation, high quality, functional flexibility, and better convenience [3]. Therefore, in order to effectively study the role of sharing economy in promoting the transformation and upgrading of the old scattered community life service industry to the innovative community life service industry and promoting the rapid development of the innovative community life service industry, it is necessary to deeply explore the structural characteristics and dynamic mechanism of the commercial network of community life service industry. Thus, through the understanding of the essence of commercial network of community life service industry, it can provide theoretical guidance and decision-making basis for the development of commercial network of community life service industry.

RETRACTED

## 2. Related Work

Liu et al. briefly analyzed the important opportunities provided by the “wisdom community” for community cooperative governance and comprehensive service system construction in ethnic minority areas, and an integrated model for the construction of a “culture sharing cloud system,” “public cultural service microplatform,” and “interactive end of public cultural service” is proposed [4]. Dong et al. focused on the analysis of the impact of network node centrality and hierarchical structure control on the network and then extended the research results of undirected network to directed network, multilayer network, and other networks [5]. Delanoy and Kasztelnik used the random walk method to divide the community of the network and brought the community division and important node mining into the analysis index of complex network structure. In recent years, the research on complex networks is more inclined to specific research in specific fields [6]. Dai et al. established the pipeline pressure information network model by using the complex network theory, identified the pipeline flow pattern by analyzing the changes of network structure parameters, and then identified the operation of the pipeline [7]. Mikalef et al. analyzed and calculated the basic node information of complex networks and found that spectrum sequence can be used to reveal the randomness and complexity of network structure, which provides a new perspective for studying and understanding the structure and function of complex networks [8]. Skolik et al. established a model of energy trade mode by combining target regression analysis and complex network and created country risk indicators to analyze the impact of country risk on energy trade mode [9]. Baskin et al. studied biological network, Internet, and local area network, respectively, and analyzed the evolution dynamics of complex networks in biological network, Internet, and local area network in detail [10]. Pilozzi et al. specifically analyzed the network evolution characteristics of Tianjin Rail Transit Network [11]. Feng et al. conducted complex network modeling for multilevel supply chain and then analyzed the robustness of cascading failures in the evolution process [12]. Höhn et al. focused on the micro behavior and characteristics of nodes in the evolution process of complex networks, affected the selection of edge to target nodes through the propagation activities and node applicability between source nodes and target nodes, and established a network evolution model [13].

RETRACTED

By introducing the idea of neural network, Peters et al. proposed a neural network model for processing graph structure data input, which is called gorignn. Therefore, they created a deep neural network model based on spatial method [14]. After that, He et al. proposed a hierarchical deep neural network for the shortcomings of gorignn model. By integrating the original data and the state information calculated by the previous layer in the cascade as the input of each layer, the problem of long-term dependence of gorignn model can be solved [15]. Höpken et al. put forward the “graph network” framework through three update functions and three cumulative functions, with the input and output constituting a graph block, and realized the classic deep neural network model, which was extended in the graph network framework, and then realized the unification of all spatial based deep neural network models in its framework. The key idea of the deep neural network model based on the spectrum theory is to use the spectrum theory to generate the graph Laplacian matrix and then extract the information propagation mechanism on the graph [16]. Auerbach and Hassett introduced the idea of spectral graph theory, proposed a new neural network model for processing graph structure data input, called spectral depth network (spectral GCN), and created a deep neural network model based on spectral graph theory [17]. Avci et al. proposed deep network (GCN) on the basis of ChebNets model [18]. Johnson and Khoshgoftaar proposed the structure depth network embedding (SDNE) model based on the idea of sparse self-encoder [19]. Andreassen et al. proposed graph recurrent neural network based on the idea of recurrent neural network. The graph recurrent neural network model mainly constructs two recurrent neural networks: one is used to generate new nodes and the other is used to add edges to new nodes in the form of autoregression [20]. Geist et al. proposed a traffic flow forecasting model based on deep neural network by combining spatial dependence modeling with time dependence modeling [21]. A session aware recommendation (mgsp) model was proposed based on multidepth neural network to solve the problem that the session-based recommendation algorithm mainly relies on the information in the target session and does not make full use of the collaborative information in other sessions.

It can be seen from the above research status that scholars have done a lot of research on complex network, community life service industry, link prediction, and deep neural network, which has laid an important research foundation for the research of this paper on the business network of community life service industry [22]. Link prediction method has been well developed in the computer field as a solution to the prediction problem in data mining. Through the research status of link prediction algorithm, we can know that link prediction algorithm has developed from the link prediction algorithm based on similarity to the link prediction algorithm based on maximum likelihood and then to the latest link prediction algorithm based on machine learning [23]. In the latest link prediction algorithm based on machine learning, the main factor restricting its development is the extraction of network features. How to better extract network structure features is the difficulty of link prediction development at this stage [24]. In recent years, the neural network in the field of image recognition has an excellent performance in extracting image features, and the deep neural network has also been better developed [25]. Therefore, the deep neural network can be used in the current link prediction field to solve the problem that the network features cannot be better extracted in the current link prediction field. However, the current research in this area is still very scarce.

RETRACTED

## 3. Domain Ontology Construction of Community Life Service Industry Sharing Economy Based on Deep Neural Network

### 3.1. Ontology Topology of Community Life Service Business Network Sharing Economy

Each node in Figure 1 represents a commercial enterprise in the community life service industry. Different companies in the network use different numbers to distinguish them. The data in the table represents the node attribute information of the community life service business network and node companies in the area, and the network topology diagram shows the network structure information of the community life service business network in the area. From the data, we can see that the information provided by the commercial network of community life service industry and the node attributes of node enterprises in the region is quite limited, and it cannot solve the problem only by relying on this limited node attribute information. Therefore, it is necessary to conduct data mining on the network structure of the commercial network of community life service industry in this region, so as to provide data information support for the later evolution of the commercial network.

### 3.2. Index Parameters of Ontology Business Network Structure Model in the Field of Sharing Economy of Community Life Service Industry

Under the framework of comprehensive analysis of ontology business network structure in the field of sharing economy of community life service industry, there are also many network structure parameter indexes of ontology business network in the field of sharing economy of community life service industry. The main indexes are as follows:

① Average degree: degree refers to the number of neighbors of a network node. The average degree is the average value of all nodes. The average degree is the analysis index of the commercial network structure of the community life service industry at the macro level, and its calculation formula is (1): the average degree is the average value of all nodes.
  (1) $$\begin{array}{c} \langle k\rangle =\frac{1}{N}\sum_{i=1}^{N}k_{i}. \end{array}$$
② Degree distribution: degree distribution refers to the probability distribution of degree value of nodes in the network, that is, the probability of nodes with degree value of *K* randomly selected from the network. Degree distribution is a macro analysis index of commercial network structure of community life service industry, and it is also an important index to judge whether the network is a classic complex network model.
③ Network density: network density refers to the density of the number of connected edges in the network. The more the edges are connected, the higher the network density is. Network density is also an analysis index of the macro level of the commercial network structure of community life service industry:
  (2) $$\begin{array}{c} \text{d}\left(G\right)=\frac{2M}{\left[N\left(N-1\right)\right]}. \end{array}$$
④ Average path: the average path is the average number of intermediate nodes that the network needs to pass through. If the average path is very small, it means that the network is easy to reach and efficient. The average path is an analysis index of the commercial network structure of the community life service industry at the macro level and also an index reflecting the efficiency of the supply chain:
  (3) $$\begin{array}{c} L=\frac{1}{n\left(n-1\right)}\sum_{i\neq j}d_{ij}. \end{array}$$
⑤ Average agglomeration coefficient: the average clustering coefficient refers to the average probability that two nodes connected to the same node are also connected to each other. The average agglomeration coefficient is the subindex of the commercial network structure of community life service industry:
  (4) $$\begin{array}{c} c_{i}=\frac{1}{k_{i}\left(k_{i}-1\right)}\sum_{j\neq k}\partial_{ij}\partial_{ik}\partial_{jk}. \end{array}$$
⑥ Community structure: community structure refers to the community formed by the close aggregation of links among nodes in the network. Community structure is an important analysis index in the meso level of the commercial network structure of community life service industry. On the one hand, it can reflect the network partial structure characteristics such as the connection preference between node enterprises and factions and small groups in the commercial network structure of community life service industry. On the other hand, it can also distinguish different types of life services in the community life services business network topology. This paper uses the Louvain algorithm, the main idea of which is to divide the community through continuous iteration, so as to make the index modularity of judging whether the community is good or bad reach the highest.

In Step 1, each node is divided into the communities where its adjacent nodes are located, and the modularity value of the current community is calculated. The modularity calculation formula is as follows:

(5) $$\begin{array}{c} Q=\frac{1}{2M}\sum_{i,j}\left[\left(\alpha_{ij}-\frac{k_{i}k_{j}}{2M}\right)\delta \left(\sigma_{i},\sigma_{j}\right)\right]=\sum_{c}\left[\frac{\sum_{\text{in}}}{2m}-\left(\frac{\sum_{\text{tot}}}{2m}\right)\right]. \end{array}$$

In Step 2, it is to reconstruct the network from the community structure divided in Step 1.

RETRACTED

In Step 3, repeat Step 1 for iteration, and maximize the modularity until the modularity no longer changes.

### 3.3. Link Prediction Algorithm for Commercial Network of Community Life Service Industry Based on Deep Neural Network

The previous summary mentioned that the biggest factor restricting the application of link prediction algorithm based on machine learning is the extraction of network features. With the development of computer vision technology, image recognition technology is more and more perfect. Convolutional neural network (CNN) has shown its unique advantages in extracting image features, so we want to use convolutional neural network in the field of link prediction to extract network features. Because the data structures of the two are different, spectral graph theory is introduced to solve this problem, and the non-Euclidean structure of graph is transformed into Euclidean data structure of matrix in order to achieve the feature extraction of the data in this paper.

The following introduces the principle of deep neural network in the community life service business network implementation process.

Firstly, the commercial network of community life service industry is described as a graph *G*=(*V*, *E*) composed of edge set *E* and point set *V*. Let the adjacency matrix of commercial network *g* of community life service industry be *a*, and the element *A*(*i*, *j*) of column *j* in row *i* of the matrix is the weight of edge (*i*, *j*). The degree matrix *D* of commercial network *g* of community life service industry is defined as follows:

(6) $$\begin{array}{c} D\left(i,i\right)=\sum_{j=1}^{n}A\left(i,j\right). \end{array}$$

The symmetric normalized Laplacian matrix of commercial network *g* of community life sex service industry is as follows:

(7) $$\begin{array}{c} L=I-D^{-\left(1/2\right)}{\text{AD}}^{-\left(1/2\right)}. \end{array}$$

The Fourier transform of the graph signal of the commercial network of community life service industry is as follows:

(8) $$\begin{array}{c} \hat{X}\left(\lambda_{i}\right)=\langle X,U_{i}\rangle =\sum_{i=1}^{n}X\left(i\right)U_{i}\left(i\right). \end{array}$$

The inverse Fourier transform of the graph signal of the commercial network of community life service industry is as follows:

(9) $$\begin{array}{c} X\left(i\right)=\sum_{i=1}^{n}\hat{X}\left(\lambda_{i}\right)U_{i}\left(i\right), \end{array}$$

where *u*_*l*_(*i*) is the *i-th* component of vector *u*_*l*_.

RETRACTED

Therefore, in the field of analog signal processing, the convolution in the time domain is equal to the inverse Fourier transform of the product of the signal in the frequency domain.

The commercial network depth of community life sex service industry can be defined as follows:

(10) $$\begin{array}{c} \left(x*\vartheta y\right)\left(i\right)=\sum_{i=1}^{n}\hat{x}\left(\lambda_{1}\right)\hat{y}\left(\lambda_{1}\right)u_{i}\left(i\right), \end{array}$$

where *∗ϑ* refers to the depth of commercial network of community life service industry. The graph signal of commercial network of community life service industry is filtered in frequency domain by using filter:

(11) $$\begin{array}{c} x*\vartheta y=U\left(\begin{array}{ccc} \hat{y}\left(\lambda_{1}\right) & \ldots & 0\\ \vdots & \ddots & \vdots \\ 0 & \ldots & \hat{y}\left(\lambda_{n}\right) \end{array}\right). \end{array}$$

This is the basic principle of deep neural network and the practical process of deep network principle in the commercial network of community life service industry. The deep network model includes several convolution layers, the input is the node attribute matrix *X*_*P*_ of *n* × *d*_*p*_ in the commercial network of community life service industry, and the output is the node attribute matrix *X*_*P*+1_ of *n* × *d*_*p*+1_ in the commercial network of community life service industry. The detailed formula is as follows:

(12) $$\begin{array}{c} X_{p+1}\left(:,j\right)=\sigma \left(\sum_{i=1}^{d_{p}}V\left(\begin{array}{ccc} \left(\overset{j}{\underset{i}{\theta }}\right)\left(1\right) & \ldots & 0\\ \vdots & \ddots & \vdots \\ 0 & \ldots & \left(\overset{j}{\underset{i}{\theta }}\right)\left(n\right) \end{array}\right)V^{T}X_{p}\left(:,i\right)\right),\forall j=1,\ldots ,d_{p+1}. \end{array}$$

In the above formula, *X*_*P*_(:, *i*) and *X*_*P*+1_(:, *j*) represent the *i* input graph signal and the *j* output graph signal of the commercial network of community life service industry, respectively. *θ* is the filter parameter vector to be learned in the commercial network model of community life service industry. The column vector of *V* is the eigenvector of *L*, and *σ* is the activation function. This is the realization of the deep neural network in the commercial network of community life service industry. The basic principle of the deep neural network is simply to say that the convolution in the time domain is equal to the Fourier inverse change of the product of the signal in the frequency domain in the analog signal processing discipline, and the convolution in the graph domain (non-Euclidean data structure) is equal to the Fourier inverse change of the product in the spectral domain (Euclidean data structure). Next, we will further elaborate the implementation process of link prediction algorithm based on deep neural network.

RETRACTED

The principles of deep neural network and convolution neural network are basically similar, but the difference lies in the different types of data. It needs to use the spectrum theory to transform the non-Euclidean structure data of graph data into the Euclidean structure data of matrix. Therefore, it needs to extract the adjacency matrix of community life service business network *G*. According to the ratio of 9 : 1, the data is separated into training data set and test data set. The separated test data set is called positive data set, and the same number of negative data sets is constructed. The negative data sets are mainly the data sets that have not been connected in the network. The test data constructed in this way is to calculate the *AUC* index, and the *AUC* formula is as follows:

(13) $$\begin{array}{c} \text{AUC}=\frac{\sum {\text{pred}}_{\text{pos}}-{\text{pred}}_{\text{neg}}}{\text{positiveNum}\times \text{negativeNum}}. \end{array}$$

Because the number of nodes in the commercial network of the community life service industry is 2375, the input adjacency matrix of the convolution layer is a 2375 ^*∗*^ 2375 matrix. In the follow-up convolution operation, the computing burden of the computer is heavy. Through the observation of the data characteristics, it is found that there are more zeros in the matrix, which belongs to sparse matrix. Therefore, the sparse matrix coding is introduced to reduce the computing burden of the computer and speed up the program. CSR coding is used here. CSR coding needs three kinds of data to express: numerical value, column index, and row offset. The numeric array stores all nonzero elements, the column index group stores the column subscripts of all nonzero elements, and the row offset array stores the row subscripts of all compressed nonzero elements.

RETRACTED

The neural network in this paper mainly consists of two layers. The input dimension of the first layer is 2375, the output dimension of the first layer is 250, and the activation function of the first layer is ReLU function. The input of the second layer is equal to the output dimension of the first layer, which is 250, the output dimension of the second layer is 25, and the second layer has no activation function. It can be seen that the neural network framework used in this paper is relatively simple. The reason is the difference between deep neural network (GCN) and ordinary convolutional neural network (CNN). Ordinary convolutional neural network needs a better and more complex neural network framework to further optimize the neural network and extract data features. However, increasing the complexity of neural network framework will only increase the burden of network operation, and the gain of neural network in feature extraction is limited. Therefore, according to the actual situation, the neural network framework with relatively simple structure is finally used.

In Step 1, put the processed data into the neural network for training:
  (14) $$\begin{array}{c} H^{\left(i+1\right)}=\sigma \left({\tilde{D}}^{-\left(1/2\right)}\tilde{A}{\tilde{D}}^{-\left(1/2\right)}H^{\left(l\right)}W^{\left(l\right)}\right), \end{array}$$
where $\tilde{A}$ is the adjacency matrix of commercial network *G*, $\tilde{D}$ is the characteristic matrix of commercial network *G*, *W* is the parameter to be trained, and *σ* is the ReLU activation function.
  (15) $$\begin{array}{c} f\left(x\right)=\max\left(0,x\right). \end{array}$$
In Step 2, each node is represented by a softmax function to get the prediction result of each tag.
  (16) Z=softmaxA˜ReLUA˜fW0Wl.
In Step 3, the expected cross entropy of all labeled nodes is taken as the loss function:
  (17) $$\begin{array}{c} \varsigma =-\sum_{l\in y_{i}}\sum_{f=1}^{F}Y_{lf}\ln\;Z_{lf}. \end{array}$$
In Step 4, the Adam optimizer is used to minimize the loss function. The deep neural network model used in this paper is shown in Figure 2. Figure 2 shows the structure diagram of the deep learning network and the transmission steps of the deep learning network.

## 4. Case Study on Ontology of Community Life Service Industry Sharing Economy Based on Deep Neural Network

### 4.1. Problem Description

Taking a large community in Beijing as an example, the permanent population of the community is about 188000, of which 28% are below 32 years, 39% are over 65 years, 65% are in families with 2-3 people, 64.2% are above college education, and 34.48% are high-income groups with 8000 yuan or more per month. The proportion of administrative office, education, finance, sports, medical, and other supporting facilities is about 30%, and the proportion of other service businesses is about 70%. In 80% of the service businesses, the retail industry accounts for 42%, and the catering industry accounts for 16%. Judging from the existing commercial formats, the community is dominated by retail industry, with the majority of large- and medium-sized high-end commercial markets and less small convenience stores.

RETRACTED

### 4.2. Ontology Simulation Experiment of Community Life Service Industry Sharing Economy Based on Deep Neural Network

The simulation experiment of this paper is based on the Python 3.7 software in Windows 10 system. The data collected in this paper are 2375 nodes, including vegetable and fruit retail, convenience store (community supermarket), catering, terminal distribution, beauty salon, and convenience maintenance, with 10523 links. Then, according to the ratio of 9 : 1, it is divided into training set and test set, and the positive and negative sample test set is constructed. The detailed process is consistent with the implementation process of the commercial network link prediction algorithm based on deep neural network, and 9472 training sets and 1052 positive and negative test sets are obtained.

Then, the data is encoded and input to the deep neural network for training. Through multiple tests, it is found that the best effect is that the number of cycles is about 650, and the change of the loss function is shown in Figure 3.

In the figure, the abscissa is the number of cycles, and the ordinate is the value of the loss function. It can be seen that the loss function tends to be calm in the continuous oscillation. The reason for the oscillation is that the mechanism of preventing overfitting is added in the process of training. The change of network final evaluation index AUC is shown in Figure 4.

As can be seen from the figure, the final AUC value of the trained model is 0.941, and the training time is 30 seconds. Thus, the link prediction model based on deep neural network is obtained. Then the link prediction model based on deep neural network is used to predict the connection between the new node and the old node. When the number of network nodes increases from 2375 to 2376, that is, the network increases, and then, according to the evolution rules of the commercial network evolution model of community life service industry and the implementation process of the link prediction algorithm of commercial network based on deep neural network, the network structure of different periods is obtained continuously. The initial network nodes of community life service industry were 2375 and they gradually evolved to 3000 nodes. Here, the simulation experiment of this paper evolves to 3000 nodes, because, through the analysis of the community life service industry in this area, when the network evolves to 3000 nodes, it basically meets the needs of the community population, and the market is basically saturated. Record the network structure of different nodes in turn, and get the following data. The topology diagram is shown in Figure 5; Figure 5 shows the needs of the community population and market saturation.

RETRACTED

The detailed data of different nodes in the network are shown in Table 1. Table 1 is a detailed description of the data in different periods, showing the development speed of the business network evolution model.

Combined with the analysis index of complex network and the quantitative analysis framework of business network of sharing economic entities in community life service industry, the following information can be obtained:

① From the increment of edge and the average increment of edge, the change of edge is shown in Figure 6. In the early period of time, the growth rate was very fast and then gradually slowed down. It was the development of Internet, Internet of things, and artificial intelligence in recent years, as well as the breakthrough of 5 g technology. Combined with the development of bike sharing and car sharing before, the breakthrough of technology, and the influx of capital, it is predicted that there will be a wave of explosive development and application of Internet of things in the next few years. Reflecting the change of network data, it is the sharp increase in the number of connected edges between 2400 and 2600 nodes. Later, the demand of technology popularization is saturated and then to a stable development, which can be seen from the gradual reduction of the average clustering coefficient. On the other hand, it is also the fact that some large Internet enterprises such as Alibaba, Jingdong, and Meituan are gradually entering into community retail, which also leads to the increase of connections between nodes to a certain extent. Enterprises like Jingdong are suppliers, distributors, and even manufacturers of some products. They can directly connect manufacturers, suppliers, and customers. From the perspective of supply chain, it is also the embodiment of optimizing supply chain structure, reducing logistics cost, and improving delivery efficiency
② From the change of average path, the average path reflects the average number of nodes from the manufacturer to the customer, as shown in Figure 7. The main reason for the decline of the average path is the development of online retail. With the popularity of online shopping, people are more and more used to online shopping. Online shopping mostly goes beyond middlemen and goes directly to customers in the mode of manufacturer direct delivery and origin direct delivery. The reason for the larger speed drop is due to the impact of COVID-19 in 2020 and online retail development. The reason why the average path is no less than 2 is that offline retail still exists, and community group buying and convenience store delivery are still the fastest and most convenient services. According to the trend of supply chain distribution cost reduction and distribution efficiency improvement, the average path should also be reduced year by year.
③ From the overall topology, it is obvious that the relationship between nodes is getting closer and closer. Through the Louvain community partition algorithm, we can get the community distribution map of the network, as shown in Figure 8. It can be seen from the figure that the middle part is closely related. By comparing the original network data, we can see that the middle part is mainly convenience stores, terminal distribution (express delivery point and express cabinet), and fruit and vegetable retail. On the one hand, with the development of community retail, the boundary between convenience stores and fruit and vegetable retail is gradually weakening. Convenience stores also sell fruits and vegetables, and fruits and vegetables also sell daily necessities. Gradually toward a community comprehensive small supermarket development, at the same time, some convenience stores also bear the function of express point. On the other hand, online retail enterprises gradually develop to offline, such as the emergence of Jingdong fresh food and hippo fresh food. Offline enterprises gradually develop online, such as convenience store delivery and community group buying. The combination of online and offline community retail makes the middle part of the network more and more closely connected. In the periphery of the network topology, we can see that several parts are relatively independent. In the network community division diagram, we can clearly see that, compared with the original network data, the most independent part is catering, followed by beauty salon and community maintenance. There is no obvious node growth in the three parts but only the increase of the connection with other nodes, that is, the increase of the connection with other nodes. The main reason is that the demand of catering, beauty, and hairdressing is relatively saturated in the development of the community, and there will be no large-scale growth. Some are just transforming to cater to the development of the market, such as catering delivery, beauty salon group buying, and door-to-door service. Therefore, the performance in the network is due to the increase of external connections.

RETRACTED

## 5. Conclusion

This paper proposes a link prediction algorithm based on deep neural network, which improves the accuracy of feature extraction of commercial network of community life service industry. Link prediction algorithm is an algorithm to predict the edges between nodes in the evolution process of complex network. It is an algorithm to process non-Euclidean data with graph as data. It is essentially different from the neural network algorithm which mostly processes Euclidean data with matrix as data at present. Therefore, the development is relatively slow for a long time. However, a difficult problem restricting its development is the extraction of network structure features. In recent years, based on the rise of deep neural network, it shows its advantages in processing non-Euclidean structured data represented by graph data and draws the public's attention to deep neural network. Therefore, deep neural network has developed rapidly. This paper studies the application of the latest deep neural network algorithm in link prediction of commercial network in community life service industry. Furthermore, it solves the problem that the current link prediction algorithm has low accuracy in network structure feature extraction.

## Figures and Tables

**Figure 1:** Display of model data construction.

**Figure 2:** The architecture of deep neural network.

**Figure 3:** Change of loss function.

**Figure 4:** Changes in AUC indicators.

**Figure 5:** Topological structure of network in different node periods.

**Figure 6:** Changes of the connection edges.

**Figure 7:** Average path length variation.

**Figure 8:** Network community structure.

**Table 1:** Detailed indicators of network evolution.

Number of nodes	Number of edges	Average degree	Network diameter	Graph density	Average clustering coefficient	Average path length
2375	10523	8.862	17	0.004	0.346	5.303
2400	11570	9.643	12	0.004	0.285	4.38
2450	14813	12.093	9	0.005	0.194	3.504
2500	17566	14.054	7	0.006	0.153	3.277
2600	21985	16.892	6	0.006	0.116	3.094
2700	24780	18.356	5	0.007	0.098	3.036
2800	26697	19.07	5	0.007	0.088	3.016
2900	28674	19.776	5	0.007	0.079	2.997
3000	30833	20.556	5	0.007	0.072	2.974

## Data Availability

The data used to support the findings of this study are available from the corresponding author upon request.

RETRACTED

## References

[1] Zheng Z. L. (2016). Research on the cause, connotation and business model of sharing economy. *Modern Economic Research*.

[2] Zhao S. D., Wang X. P. (2018). Sharing city planning strategy driven by sharing economy. *The Planner*.

[3] Fang Y., Xu H., Perc M., Tan Q. (2019). Dynamic evolution of economic networks under the influence of mergers and divestitures. *Physica A: Statistical Mechanics and its Applications*.

[4] Liu X. (2021). Intelligent integrated community model for ethnic minority areas using data analysis and machine learning. *Mobile Information Systems*.

[5] Dong J., Chen Y., Guan G. (2020). Cost index predictions for construction engineering based on LSTM neural networks. *Advances in Civil Engineering*.

[6] Delanoy N., Kasztelnik A. (2020). Business open big data analytics to support innovative leadership and management decision in Canada. *Business Ethics and Leadership*.

[7] Dai H. N., Wang H., Xu G. (2020). Big data analytics for manufacturing internet of things: opportunities, challenges and enabling technologies. *Enterprise Information Systems*.

[8] Mikalef P., Boura M., Lekakos G. (2020). The role of information governance in big data analytics driven innovation. *Information & Management*.

[9] Skolik A., McClean J. R., Mohseni M. (2021). Layerwise learning for quantum neural networks. *Quantum Machine Intelligence*.

[10] Baskin C., Liss N., Schwartz E. (2021). Uniq: Uniform noise injection for non-uniform quantization of neural networks. *ACM Transactions on Computer Systems*.

[11] Pilozzi L., Farrelly F. A., Marcucci G., Conti C. (2021). Topological nanophotonics and artificial neural networks. *Nanotechnology*.

[12] Feng R., Grana D., Balling N. (2021). Uncertainty quantification in fault detection using convolutional neural networks. *Geophysics*.

[13] Höhn J., Hekler A., Krieghoff-Henning E. (2021). Integrating patient data into skin cancer classification using convolutional neural networks: systematic review. *Journal of Medical Internet Research*.

[14] Peters E., Kliestik T., Musa H. (2020). Product decision-making information systems, real-time big data analytics, and deep learning-enabled smart process planning in sustainable industry 4.0. *Journal of Self-Governance and Management Economics*.

[15] He Z., Tang X., Yang X. (2020). Clinical trial generalizability assessment in the big data era: a review. *Clinical and translational science*.

[16] Höpken W., Eberle T., Fuchs M. (2021). Improving tourist arrival prediction: a big data and artificial neural network approach. *Journal of Travel Research*.

RETRACTED

[17] Auerbach A. J., Hassett K. (2017). Optimal long-run fiscal policy: constraints, preferences and the resolution of uncertainty. *Journal of Economic Dynamics and Control*.

[18] Avci C., Tekinerdogan B., Athanasiadis I. N. (2020). Software architectures for big data: a systematic literature review. *Big Data Analytics*.

[19] Johnson J. M., Khoshgoftaar T. M. (2020). The effects of data sampling with deep learning and highly imbalanced big data. *Information Systems Frontiers*.

[20] Andreassen A., Hsu S. C., Nachman B. (2021). Parameter estimation using neural networks in the presence of detector effects. *Physical Review D*.

[21] Geist M., Petersen P., Raslan M. (2021). Numerical solution of the parametric diffusion equation by deep neural networks. *Journal of Scientific Computing*.

[22] McKinley R., Wepfer R., Aschwanden F. (2021). Simultaneous lesion and brain segmentation in multiple sclerosis using deep neural networks. *Scientific Reports*.

[23] Gui G., Zhou Z., Wang J., Liu F., Sun J. (2020). Machine learning aided air traffic flow analysis based on aviation big data. *IEEE Transactions on Vehicular Technology*.

[24] Surbakti F. P. S., Wang W., Indulska M. (2020). Factors influencing effective use of big data: a research framework. *Information & Management*.

[25] Kend M., Nguyen L. A. (2020). Big data analytics and other emerging technologies: the impact on the Australian audit and assurance profession. *Australian Accounting Review*.

